The article "Teachers' Teaching Ability Promotion Strategies Based on Lightweight Deep Learning Combined with Target Detection Algorithm" was retracted in 2023. Reasons: signs of a paper mill; suspected computer-generated content; unreliable results or conclusions; concerns about the data.

# Teachers' Teaching Ability Promotion Strategies Based on Lightweight Deep Learning Combined with Target Detection Algorithm

**DOI:** 10.1155/2022/4880560

**Published:** 2022-07-12

**Authors:** Yuqian Jin

**Affiliations:** Department of Faculty Affairs & Faculty Development, Xi'an Technological University, Xi'an, Shaanxi 710072, China

## Abstract

With the popularization of standardized classrooms in colleges and universities, it is possible to collect video data of students' class status through the camera device in the classroom. With abundant video data sources, it is easy to obtain big data of students' class status images. Unstructured video big data is a topic worthy of research in improving teaching quality. First, the current teaching ability of teachers in colleges and universities is investigated, and its problems are found. Then, the You Only Look Once (YOLO) network in the object detection network is mainly studied. The deficiencies in the network structure are further explored and optimized. It is used in real classroom scenarios as well as on student expression detection problems. Finally, the proposed scheme is tested. The test results show that at present, 20% and 38% of teachers in higher vocational colleges think that they are “dissatisfied” with their classroom teaching and practical guidance ability. And 38% of teachers wanted to improve the bad situation. The accuracy of the proposed model for student expression detection is higher than that of faster-region convolutional neural network and mask-region convolutional neural network by more than 8%, higher than the YOLO v3 model by more than 4%, and higher than YOLO v3 Tiny model above 6%. The proposed model provides some ideas for the application of deep learning technology in the improvement of teachers' teaching ability.

## 1. Introduction

Since the twenty-first century, countries worldwide have come to realize the importance of higher education teaching quality. With the rapid socioeconomic and industrial structural revolution, talents have become the core competency in many industrial sectors. Thus, colleges and universities (CAUs) are expected to cultivate more industry-specific, application-ready, and innovative graduates who are the main powerhouse of social and economic advancement. In particular, the tenet of “Internet +” is prevailing swiftly, and “mass entrepreneurship and innovation” is deeply rooted in people's hearts. The “craftsman spirit” has become the professional soul of skilled talents. Society as a whole has actively strengthened the cooperation, innovation, creativity, and professional spirit of laborers. Working at the forefront, teachers in higher vocational colleges (HVCs) directly affect the quality of personnel training [1]. Therefore, it is of great practical significance to study the teaching ability promotion (TAP) strategies of HVC teachers from the perspective of teacher-student cooperation (TS-C) [2]. At the same time, intelligent science and technology (S&T) contributes considerably to the national economy and social well-being. From the perspective of higher education, the artificial intelligence (AI) S&T major is the basis for cultivating “intelligent” talents. The setting of first-level disciplines for AI S&T majors is also imminent. Convolutional neural networks (CNNs) have caught the eyes of many scholars in deep learning (DL) because of their excellent performance in image recognition (IR), natural language processing (NLP), and many other AI applications [3–5].

Researchers have conducted sufficient work in related fields. Lai et al. [6] claimed that teachers' teaching performance differed significantly. They surveyed 209 German mathematics teachers and 4,672 students. Standardized tests and self-reporting evaluated teachers' cognitive ability, personality characteristics, professional knowledge, teaching belief, and enthusiasm. The findings indicated that extraversion, teaching enthusiasm, and teaching/psychological knowledge were key metrics of learning support. Teaching conscientiousness and teaching enthusiasm were significant classroom metrics for discipline. Liu et al. [7] observed that available students' psychological research has concentrated on their and their teachers' perceptions of intellectual plasticity. However, teachers' mindsets about the plasticity of their own teaching abilities and how these teaching mindsets shaped their motivation and engagement have been rarely explored. Accordingly, the research used teachers' teaching motivation to estimate teachers' work engagement. The results suggested that a growth teaching mindset positively forecasted autonomous motivation, which in turn predicted higher work engagement. Mallaeva [8] supported flipped teaching in CAU by interacting with motivational factors, self-efficacy, and flipped teaching resources. They investigated 169 CAU teachers and revealed that intrinsic challenge motivation and extrinsic compensation motivation are the significant forerunners of teachers' willingness to use flipped teaching. Yusupjanovna [9] reasoned that in the Internet era, information-based teaching has become the most basic and critical ability of teachers for applying advanced information technology (IT) in education. They researched the teacher-oriented preservice training (PST) from three aspects: PowerPoint (PPT) skills, multimedia courseware production, and micro-lectures. The study found that integrating multimedia courseware production enriched information-based teaching resources and micro-lectures enhanced students' evaluation of teachers' information teaching. To sum up, despite their contributions, there are still some deficiencies in existing works. For example, teacher-student cooperation is now a significant theme in improving learning efficiency and teaching effect. However, few studies have involved TAP from the perspective of TS-C. Second, to improve the quality of HVC teachers, foreign research focuses on the vocational training of teachers and the leading role of enterprises. Domestic research stresses the deep cooperation between schools and enterprises and the path of deepening the production-education integration based on international experience. However, both have ignored the in-depth research on teachers' professional development through the deep integration of production and education.

At present, the education industry has entered the era of intelligent application development. The intelligent realization of students' classroom behavior recognition must put forward higher standards and requirements for students' classroom behavior analysis. In the process of building a smart campus, the classroom teaching mode should be combined with the development of the times and should not be limited to the original inherent mode. Based on the current situation and challenges, colleges and universities have established analysis systems for classroom teaching activities to complete the intelligent research in teaching. In recent years, with the rapid development of artificial intelligence, advanced science and technology can not only break the constraints of time and space and innovate the way of classroom teaching but also improve the atmosphere and efficiency of classroom teaching activities and further accelerate the pace of smart campus construction. From ancient times to the present, although China's education system has been reformed, there are still some imperfections. Classroom teaching analysis is an important way and a key link in the reform of the education system. As the main content of classroom teaching analysis, the identification of students' behavior status, its rationality, and effectiveness will have a direct impact on the teaching effect. Comprehensive observation and reasonable statistics of students' behavior in the classroom will help to evaluate and adjust the way, content, and focus of teachers' teaching. Additionally, the construction of smart campus will also develop steadily. The recognition of students' classroom behavior status by target detection algorithm not only highlights the educational concept of contemporary society but also realizes the combination of deep learning theory and classroom teaching activities. However, with the continuous innovation of target detection algorithms and the complexity and change of classroom scenes and student behaviors, the existing algorithms can no longer meet the needs of the current smart campus construction, especially in the accuracy of students' classroom behavior status recognition. The innovation of target detection algorithm is far behind the pace of smart campus construction. Therefore, in order to rapidly combine the deep learning theory with the application of education and teaching, realize the intelligentization of classroom teaching and promote the construction and development of smart campus, this study is of great significance to study the state identification of students' classroom behaviors based on CNNs. Based on the above literature review, this paper studies the teachers' TAP strategies based on DL from the perspective of TS-C. The innovations can be explained from two points. The first point is to uncover the existing problems in CAU teachers' teaching activities and put forward suggestions and countermeasures. The other point is to learn from the lightweight network MobileNetv2 and introduce depthwise separable convolution (DSC) and a linear bottleneck structure with inverted residuals.

The research is unfolded as follows.  Section 1 gives an overview of the current situation of teachers' TAP and the application of DL technology in TAP.  Section 2 investigates the teachers' teaching ability in a college and proposes optimization strategies. Then, Section 3 studies the target detection algorithm (TDA), the YOLOv3 model, and proposes an improved YOLOv3 model. The experimental results are analyzed in Section 4. Lastly, Section 5 summarizes the full text and explains the shortcomings and prospects for future research directions.

## 2. Research on Teachers' TAP

### 2.1. The Current Situation of CAU Teachers' Teaching

In order to understand the current situation and existing problems of teachers' teaching abilities, this paper selects full-time teachers in an HVC in XX Province. The teachers' teaching ability is analyzed by referring to related literature in HVC. A Questionnaire Survey (QS) is conducted. Overall, 210 QSs are distributed, and 153 are recovered, with a recovery rate of 72.8%. Then, 43 invalid QSs are excluded, leaving 110 valid ones, with an effective recovery rate of 52.3%.

The basic situation of the QS subjects is shown in Figure 1:

In Figure 1, the teaching qualifications of the surveyed teachers are in line with the requirements of teaching staff construction in HVCs. Thus, TAP has become the top priority in the current teacher development in the HVC. Apparently, the subjects are mainly young and middle-aged teachers with strong learning acceptance and great development potential. It is easier to form a learning team organization.

### 2.2. Existing Problems in Teachers' Teaching Ability

Analyzing the QS results has uncovered some problems in the HVC teachers; teaching abilities. (1) Insufficient motivation and emphasis on academic research over teaching activities are common in HVCs and the daily work status of teachers. Such teaching management and evaluation systems weaken the teaching efforts of front-line teachers, depriving teachers of the sense of belonging (SoB) and security in the school organization. Besides, academic research has become the primary job of HVC teachers. The “difficulty in publishing teaching and research papers” has discouraged teachers from dedicating themselves to teaching activities. Inevitably, teachers' awareness of professional development is weakened, and they become less motivated in teaching. (2) Lack of cooperation. According to the QS, HVC teachers rarely implement collaborative teaching, cooperative research, and interactive reflection with colleagues in the school, and 80% of teachers' cooperation is accidental behaviors. (3) At present, the teaching force of HVCs is characterized by a younger generation with excellent educational backgrounds. Most teachers are in the growth stage, and their teaching ability is not yet mature. It is still an essential part of the growth of young teachers to effectively and scientifically transform the broad professional knowledge and vocational skills theory into teachers' practical ability.

## 3. DL and Lightweight Object Detection Networks

### 3.1. DL Technical Analysis

There have been many major breakthroughs in DL technologies, such as Stanford University's parallel computing platform with 16,000 central processing unit (In 2012) cores proposed in 2012 [10–12]. The platform was called deep neural network (DNN). To illustrate another, in 2016, scholars designed a DL-based artificial Go software that successfully challenged the world's top Go master Lee Sedol successfully. This event marks the boom of DL Research and Development (R&D). ML explores ways to simulate or realize the intelligent beings' learning behaviors by the computer to acquire knowledge or skills, modify existing data structures, and enhance program performance. From a statistical point of view, ML predicts data distribution, learns a model from the given data, and then uses this model to estimate new data. Notably, the test and training data in the ML process must follow the same distribution [13, 14]. In other terms, ML imitates the information processing pattern of neurons in the brain. So far, ML applications are very successful in computer vision (CV) and NLP. Since DL and neural neuron (NN) are strongly correlated, DL is sometimes referred to as improved NN. In the modern sense, the deep CNN (DCNN) originated from the AlexNet [15, 16]. Compared with the previous CNNs, DCNN has the starkest feature: deeper layers are deepened and more complex parameters. The DCNN structure is drawn in Figure 2:

### 3.2. TDA and Lightweight CNN

TDA development can be divided into two periods: the traditional TDAs (1998–2014) and the DL-based TDAs (2014-present). The DL-based TDA has developed into two technical routes: the anchor-based method and the anchor-free method. The traditional TDA is based on manual feature extraction (FE), unlike the CNN with automatic feature extraction (FE) ability. First, the traditional TDA flow can be summarized as follows: (1) select the region of interest and select the object-hotspot region. (2) Perform FE on object-hotspot regions. (3) Detect and classify the extracted features. Traditional TDAs based on manual-extracted features have slow progress and low performance. It was not until 2012 that the rise of CNN pushed the field of object detection to a new level [17, 18]. There are two main technical development routes for CNN-based TDAs: anchor-based and anchor-free methods. Anchor-based methods include one-stage and two-stage detection algorithms.  Figure 3 portrays the TDA flow.

In Figure 3, the task of object detection is to find all objects of interest in an image and determine their category and location. These tasks are one of the core problems in the field of computer vision. Object detection is also a challenging task in computer vision due to the different appearances and shapes. It poses various objects, coupled with the interference of factors such as illumination and occlusion. In machine vision, there are four categories of tasks for object detection. Classification is the goal of judging what category is contained in a given image or a video. Positioning can find the location of this target. Detection is to find the location and object of the target. Segmentation is divided into the instance and scene segmentation to solve the problem of the attribution of each pixel object or scene.

The traditional object detection algorithm is divided into three main steps, namely region proposal, feature extraction, and classification regression. The region proposal is to traverse the image multiple times through sliding windows of different scales to obtain the region where the object of interest may be, that is, the candidate region. Feature extraction uses artificial feature extraction to convert the image in the candidate area into a feature vector, common methods such as local binary pattern features, gradient histogram features, etc. Classification and regression use a pretrained classifier to predict the class of objects in the candidate region. The disadvantage is that the traditional target detection algorithm has many redundant computations in the region proposal and can only extract low-level features during feature extraction. The whole process is divided into three stages. The algorithm cannot find the optimal global solution.

Since the invention of AlexNet in 2012, CNN has been widely used in image classification, image segmentation, and target detection. With the increasing performance requirements, AlexNet has not met practical needs. Thus, a myriad of high-performance CNNs have been proposed, such as Visual Geometry Group (VGG), GoogLeNet, Residual Network (ResNet), and Densely Connected Network (DenseNet). Meanwhile, better performance often means deeper layers, from seven-layer AlexNet to 16-layer VGG to 22-layer GoogLeNet to 152-layer ResNet to thousands of layers of ResNet and DenseNet. As a result, the trade-off between performance and efficiency must be considered. Recently, researchers have focused on engineering techniques, such as model light-weighting and compression [19, 20], resulting in several practical models: SqueezeNet, MobileNet, and ShuffeNet. The lightweight model chooses the bottleneck structure, grouped convolution structure, and small size convolution kernel. The link pattern of a common CNN is presented in Figure 4:

In Figure 4, the method is also the most standard neural network linking method. Since LeNet was proposed, the layer-by-layer linking method has been the mainstream design method. The most typical example is the Visual Geometry Group Net (VGGNet) that appeared in the ImageNet competition. The convolution calculation is performed according to the size of the feature map stage by stage, and the same convolutional layers are stacked in the same stage. The biggest feature of this linking method is that it is neat, and there are also big problems. As the depth increases, the training becomes more and more difficult, and problems such as gradient dispersion and nonconvergence appear.

### 3.3. YOLO CNN

The DL-based TDA mainly includes the region CNN (R-CNN), the single shot multibox detector (SSD), and faster R-CNN. The faster R-CNN features a high target detection accuracy, only with a prolonged processing time. Though faster R-CNN outmatches R-CNN, it is dimmed by SSD and YOLO in terms of speed [21]. With careful consideration, the YOLO is the most practical and prevailing TDA, with both fast detection speed and high detection accuracy. YOLO has several versions: v3, v4, and v5. The present work selects YOLOv3 for detecting objects from student pictures [22, 23]. The basic structure of the YOLOv3 and the tiny YOLO are illuminated in Figures 5 and 6, respectively.

YOLOv3 is mainly composed of Conv-BN-Leaky Relu (CBL), RES, and CONCAT modules. The CBL module is the basic component, including a convolutional layer, a batch normalization (BN) layer, and a leaky-relu. The number behind the RES module indicates the number of res units. CONCAT is tensor splicing, which splices the middle layer of darknet and the upsampling of the last layer. The darknet-53 is the backbone network of YOLOv3 and outputs three feature maps of different scales, that is, 13 ∗ 13 ∗ 225, 28 ∗ 28 ∗ 225, and 52 ∗ 52 ∗ 225. More delicate objects can be detected through multiscale target detection.

The Tiny YOLOv3 removes the last few layers of the MobileNetV3 and only retains all the previous blocks containing convolutional layers to replace the original DarkNet-53 network in YOLOv3. At training time, the network receives images with a resolution of 416 pixels × 416 pixels. Tiny YOLOv3 extracts feature images of the 73rd layer (52 × 52 pixels), the 135th layer (26 ×26 pixels), and the last layer (13 × 13 pixels) to complete the detection task. The feature map of 13 pixels × 13 pixels is transformed into the number of channels through 1 × 1 convolution and 3 × 3 convolutions, and the first prediction result is output. Additionally, the predicted results are upsampled to 38 pixels × 38 pixels, and the output results of the 135th layer are fused. After changing the number of channels, the second result is output. Similarly, the third prediction result is obtained. The three results are concatenated as the final prediction result.

### 3.4. Lightweight YOLO Modeling

In order to realize lightweight YOLOv3, this paper replaces its backbone with lightweight ShuffleNetv2. Then, the low-level and middle-level features output by ShuffleNetv2 are transformed, splicing them into high-level features. As such, it enriches the feature representation. The multiscale features are fused by upsampling, and the multiscale detection and the fusion of the corresponding results are used to finally realize the fast and accurate recognition of students' expressions. The improved lightweight YOLO v3 uses ShuffulNetv2 as the backbone and contains three different scale feature maps (stage2, stage3, and stage4). The input image has undergone multiple convolutions of stage2, stage3, and stage4, and after pooling, the feature size is only 12 × 12.

The linear bottleneck structure with inverted residuals can fully use smaller input feature maps and output dimensions. In order to improve the FE efficiency, the linear bottleneck module is introduced into the improved YOLOv3. The linear bottleneck module has an inverted residual structure. Point-by-point convolution is performed on a *W* × *H* × *C*, a 1×1 input feature map, and more facial expression features are obtained by expanding the channel. Then, a 3 × 3-depth convolution is performed to extract key features, and finally, a *C*_out_-channel feature map is generated through a 1 × 1 point-by-point convolution. Through the *K*_*W*_ × *K*_*h*_ convolution kernel, the input channel *C* is expanded by the expansion factor *t* to *tC*. The number of input and output channels in the middle layer remains unchanged. Then, the linear bottleneck module's computational consumption is calculated in equation (1) by ignoring the addition operation due to computational bias:

(1) $$\begin{array}{c} W\times H\times C\times t\times \left(C+K_{w}\times K_{h}+C_{\text{out}}\right). \end{array}$$

The computation ratio between the linear bottleneck structure and the DSC is counted by

(2) $$\begin{array}{c} \frac{W\times H\times C\times t\times \left(C+K_{w}\times K_{h}+C_{\text{out}}\right)}{K_{w}\times K_{h}\times W\times H\times C+1\times 1\times C\times W\times H\times C_{\text{out}}}=t\left(\frac{C}{K_{w}\times K_{h}+C_{\text{out}}}+1\right). \end{array}$$

The intersection ratio is the overlap ratio of the candidate and the marked frames. The ratio of their intersection and union is used to judge the overlap degree between the predicted frame and the real frame. Its mathematical expression reads:

(3) $$\begin{array}{c} IOU=\frac{S_{AB}\;\cap^{}S_{C\;D}}{S_{AB}\;\cup^{}S_{C\;D}}. \end{array}$$

In equation (3), *S*_*AB*_ is the marked ground-truth box, and *S*_*C*  *D*_ denotes the predicted bounding box.

The clustering algorithm [24] filters the bounding boxes. The Intersection Over Union (IOU) score is used as the final evaluation index. This method can automatically filter out suitable bounding boxes. The distance measure between the prior box and the cluster center reads:

(4) $$\begin{array}{c} D\left(B,C_{k}\right)=1-IOU\left(B,C_{k}\right). \end{array}$$

In equation (4), *B* and *B* are the predicted bounding box and *C*_*k*_ clustering center.

The product of the conditional category probability of the grid and the confidence of each prediction box is used to calculate the confidence *S*_*i*_ of each category, as expressed in:

(5) $$\begin{array}{c} \begin{array}{c} S_{i}=P\left(C_{i}|Fas\right)\cdot \mathrm{Pr}\left(Fas\right)\cdot IOU_{\text{pred}}^{\text{truth}}\\ =P\left(C_{i}|Fas\right)\cdot C_{i}. \end{array}. \end{array}$$

In equation (6), *P*(*C*_*i*_*|Fas*) is the probability that the facial expression belongs to a specific category when the grid contains the center of the face. Pr(*Fas*) represents the probability of the grid unit containing the center of the face. *IOU*_pred_^truth ^ means the IOU value of the real frame and the predicted frame of the face. *C*_*i*_ denotes the confidence of the predicted frame. The calculation of center point coordinates and size of the bounding box reads:

(6) $$\begin{array}{c} b_{x}=\sigma \left(t_{x}\right)+C_{x}, \end{array}$$

(7) $$\begin{array}{c} b_{y}=\sigma \left(t_{y}\right)+C_{y}, \end{array}$$

(8) $$\begin{array}{c} b_{w}=p_{w}e_{i}^{t_{w}}, \end{array}$$

(9) $$\begin{array}{c} b_{h}=p_{h}e_{i}^{t_{h}}. \end{array}$$

In equations (6)–(9), (*C*_*x*_, *C*_*y*_) is the upper left corner coordinate of the square containing the detected face center in the feature map. (*b*_*x*_, *b*_*y*_) represents the center coordinate of the model-predicted bounding box. (*b*_*w*_, *b*_*h*_) means the width and height of the predicted bounding box. (*t*_*x*_, *t*_*y*_) signifies each bounding box's bias abscissa and ordinate by the actual training output. (*t*_*w*_, *t*_*h*_) refers to the width and height of each bounding box by actual network training. (*p*_*w*_, *p*_*h*_) stands for the predicted width and height of the prior box.

Here, the loss function error of the proposed NN is mainly composed of three parts: center coordinate and width and height error, confidence error, and target classification error, written in:

(10) $$\begin{array}{c} \text{Loss}=L_{\text{coord}}+L_{\text{con}}+L_{\text{class}}. \end{array}$$

In equation (10), *L*_coord_, *L*_con_, and *L*_class_, respectively, represent the coordinate and width and height error, the confidence error, and the classification error between the predicted and the real bounding box.

The mathematical expression of *L*_coord_ reads:

(11) $$\begin{array}{c} L_{\text{coord}}=\lambda_{\text{coord}}\sum_{i=0}^{S^{2}}\sum_{j=0}^{B}1_{ij}^{obj}\left[s\left(x_{i},y_{i}\right)\right]+\lambda_{\text{coord}}\sum_{i=0}^{S^{2}}\sum_{j=0}^{B}1_{ij}^{obj}\left(2-w_{i}*h_{i}\right)\left[s\left(w_{i},h_{i}\right)\right]. \end{array}$$

In equation (11), *λ*_coord_ is the penalty coefficient of the coordinate error, 1_*ij*_^*obj*^ denotes the prediction frame parameter, (*x*_*i*_, *y*_*i*_) signifies the center point coordinate of the real frame, and (*w*_*i*_, *h*_*i*_) refers to the width and height of the real frame. *L*_con_ can be counted by

(12) $$\begin{array}{c} L_{\text{con}}=\sum_{i=0}^{S^{2}}\sum_{j=0}^{B}1_{ij}^{obj}f\left(C_{i},{\hat{C}}_{i}\right)+\lambda_{noobj}\sum_{i=0}^{S^{2}}\sum_{j=0}^{B}1_{ij}^{noobj}f\left(C_{i},{\hat{C}}_{i}\right). \end{array}$$

In equation (12), *λ*_*noobj*_ is the penalty coefficient of the confidence error. $\left(C_{i},{\hat{C}}_{i}\right)$ stands for the confidence error between the predicted and real the bounding box. 1_*ij*_^*noobj*^ means the *i*th grid containing the *j*th candidate frame contains no detection center. *C*_*i*_ indicates the confidence of the *i*th grid in the ground truth box. Lastly, ${\hat{C}}_{i}$ stands for the confidence of the *i* th grid in the prediction box.

The algorithm flowchart is shown in Figure 7.

### 3.5. Data Set and Model Configuration

This section uses the MMI Facial Expression Database [25], obtained by 32 participants posing for specified expressions under laboratory conditions containing 2,900 videos and 720 ∗ 576-pixel 740 images. Before the model is trained, the software YOLO Mark is used to manually label the faces in the images with the target's category and location. The coordinates of the rectangular frame are normalized to [0, 1] for the convenience of maintaining the coordinate data during data enhancement. The YOLO annotation information is stored in a text file with the same name as the image. Each line represents a target and includes five parameters: the target category number, the x-coordinate and the y-coordinate of the rectangle's center, and the rectangle's width and height.  Figure 8 sketches the experimental data set from MMI Facial Expression Database.

Model training uses graphics processing unit (GPU) server. The hardware configuration is as follows: Intel E52665X2; 32 GRECC DDR3; 250G Solid State Drive (SDD); four NVIDIA RTX 2080TI 11G graphics cards. The software is configured below like Ubuntu Linux 16.04; CUDA10.0; cuDNN7.6. The experiment is completed on a laptop computer with an Intel i79750H 4.5 GHz 6-core CPU, a 32G DDR4 2666 RAM, and a GeForce GTX 1650 GPU. The laptop is deployed with a Windows10 operating system and CUDA10.1, Cudnn7.6, and OpenCV3.4.1 software developing environment.

Model training and evaluation are based on optimized YOLOv3, using 64 samples as processing units. Batch normalization (BN) is performed every time the weight is updated. Other parameters are set as momentum = 0.9; saturation = 1.5; exposure = 1.5; initial learning rate = 0.001; the learning rate variation factor = 0.1; and the learning rate control parameter = 1,000. There is only one target category, so the maximum iteration is 4,000 times.

## 4. Results and Discussion

### 4.1. QS Reliability and Validity Analysis

Table 1 lists the reliability and validity analysis results of the designed QS.

In Table 1, in the test scale, the value of Sig. for each variable and dimension is 0.000, and the value of Kaiser-Meyer-Olkin (KMO) is greater than 0.7. The values of this scale are suitable for factor analysis. Eigenvalues greater than 1.5 are used to determine the number of common factors based on similarity. The variance explained rate is 82.34%.

### 4.2. QS Results of Teachers' Teaching Ability

Figure 9 plots the QS results of the teacher's teaching ability.

In Figure 9, the QS results display the HVC teachers' satisfaction with their teaching abilities and teaching effects. Specifically, 20% of teachers are dissatisfied with their teaching skills and 38% are dissatisfied with their practical guidance ability. Thus, most HVC teachers are satisfied with their teaching ability, with obvious demands for TAP in practical guidance. Additionally, teachers' views are consistent in teaching effects on theoretical knowledge and technical ability. All believe that their theoretical and practical abilities are equal. Based on the above data analysis, teachers believe that their teaching ability meets the requirements of higher vocational education and can qualify for talent training tasks. Second, most teachers recognize the existing problems in their teaching ability. They hope to improve their teaching ability, especially the TAP, in practical guidance.

### 4.3. DL TDA Testing

Figure 10 charts the network loss curve of the nonimprovedYOLOv3 and the proposed improved YOLOv3.

In Figure 10, in the proposed improved YOLOv3 model, from the 3,500^th^ iteration on, although the loss curves at 4,550 and 6,800 have small peaks. The overall network loss shows a downward trend and tends to be flat. From the 8,000^th^ iteration on, the network loss stabilizes below 0.2. By comparison, in the nonimproved YOLOv3 model, from the 7,800^th^ on, the network loss stabilizes below 0.25. Thus, the unimproved network always has a higher training error than the improved network. The training effect of the improved model is better than the unimproved model.

Table 2 enumerates the performance comparison of the proposed improved YOLOv3.

As shown in Table 2, the detection accuracy of the proposed improved YOLOv3 model is the highest among all models. It is more than 8% higher than the Faster R-CNN and the Mask R-CNN, 4% higher than the YOLOv3, and 6% higher than the Tiny YOLOv3 [26]. Additionally, the recall of the proposed model is higher than that of the Faster R-CNN model and the Mask R-CNN model [27]. Hence, the proposed improved YOLOv3 model can better trade-off recall and prediction accuracy.

The detection accuracy of the proposed improved YOLOv3 model for smiling and sad expressions is 4.22% and 8.6% higher than the Tiny YOLOv3 model and 5.22% and 9.6% higher than the Mask R-CNN model. Compared with other current detection networks, the proposed model has superior facial expression detection ability that is shown in Figure 11.

Table 3 compares the time complexity of different models.

As in Table 3, the FPS of the Faster R-CNN, Mask R-CNN, YOLOv3, and Tiny YOLOv3 is 2.2, 1.6, 5.8, and 23.2, respectively. The FPS of the proposed improved YOLOv3 is 14. Although the FPS of the proposed improved YOLOv3model is lower than the Tiny YOLOv3 [28, 29], the model performance is compensated by the high facial recognition accuracy mAP.

### 4.4. Algorithm Comparison

Figure 12 compares the test and training time of the proposed model and other models.

From Figure 12, the time consumed by the improved YOLOv3 model and the YOLO v4 model in the detection process is similar when testing the real scenes 1, 2, and 3. However, the gap between YOLOv4 and the improved YOLO v3 increases with the continuous data increase. In short, the proposed improved YOLOv3 model is feasible for evaluating the quality of classroom teaching in CAU.

## 5. Conclusion

The development of teachers' abilities is an important part of improving the overall quality of the profession, and it needs to be highly concerned by all parties. Therefore, deep learning techniques are used to research teacher competencies. The improved YOLOv3 algorithm is proposed to recognize students' facial expressions and let teachers change the mode of class according to the changes of their facial expressions. Experiments show that the detection accuracy of the improved network for smiling and sad expressions is 4.22% and 8.6% higher than the YOLO v3-Tiny model and 5.22% and 9.6% higher than the Mask R-CNN model. Compared with other current detection networks, the improved network model has superior expression detection ability. At present, the detection of basic categories has been initially implemented. However, at the macro-analysis level, this study still has some problems that need to be improved and further studied. The photo collection environment is relatively severe. There are problems of unstable and insufficient light during the collection process. Even if a professional industrial camera is used to capture pictures, there will be many interferences such as noise, insufficient light, and occlusion of the shooting angle. How to overcome the complex background, the occlusion of the light, and the target detection is also a direction that needs improvement. In addition, this study only selects the teaching field and initially proposes the target detection idea for the student group. However, the entire detection system still has a lot of room for improvement and further research, such as embedding computer vision into more and wider fields.

## Figures and Tables

**Figure 1:** Basic information of teachers. (in Figure 1, the meaning of the abscissa is the basic situation of the teachers under investigation. 1–16 represent the teaching age of the teachers; male and fe represent the gender; yes represents the normal class; no represents the non-normal class; other indicates others; lec means lecturer; ass means associate professor; pro means professor).

**Figure 2:** DCNN structure diagram.

**Figure 3:** The process of TDA.

**Figure 4:** Link pattern of ordinary CNNs.

**Figure 5:** YOLOv3 structure.

**Figure 6:** Tiny YOLOv3 structure.

**Figure 7:** Flow of the algorithm.

**Figure 8:** Experimental data set from MMI facial expression database.

**Figure 9:** QS results ((a) teaching ability; (b) teaching effect).

**Figure 10:** Network loss curve ((a) scene 1; (b) scene 2) (in Figure 10, the learning rate for the first test is 0.0005; the second is 0.0001; the third is 0.005; the fourth is 0.001; the fifth is 0.001 0.05; the sixth is 0.01).

**Figure 11:** Detection network test accuracy ((a) smile; (b) sadness).

**Figure 12:** Algorithm comparison ((a) scene 1; (b) scene 2; (c) scene 3).

**Table 1:** The reliability and validity of the QS.

Variable	Question	Element	Other	Variable	Question	Element	Other
1	a	0.701	(KMO = 0.821, sig = 0.000)	2	a	0.588	(KMO = 0.761, sig = 0.000)
	b	0.688			b	0.703	
	c	0.714			c	0.745	
	d	0.766			d	0.718	

3	a	0.543	(KMO = 0.766, sig = 0.000)	4	a	0.771	(KMO = 0.763, sig = 0.000)
	b	0.768			b	0.772	
	c	0.641			c	0.721	
	d	0.799			d	0.867	

(In Table 1, the meanings of a, b, c, and d are different selections in the questionnaire).

**Table 2:** Performance comparison of the improved YOLOv3.

Network model	Backbone network	F1-score	Average precision	Memory consumption
Faster R-CNN	FPN-resNet 50	0.84	90.47	495.6
Mask R-CNN	FPN-resNet 50	0.84	90.44	526.0
YOLOv3	DarkNet-53	0.9	94.22	240.6
YOLOv3 tiny	Tiny darkNet	0.81	92.47	33.1
The proposed improved YOLOv3	The designed framework	0.92	98.90	19.1

**Table 3:** Time complexity comparison of facial expression detection models.

Network model	Size of the picture	Size adjustment	Extrapolation time (ms)	Speed (FPS/frames per second)
Faster R-CNN	4096 ∗ 4096	833 ∗ 500	441.2	2.2
Mask R-CNN	4096 ∗ 4096	833 ∗ 500	618.1	1.6
YOLOv3	4096 ∗ 4096	416 ∗ 416	172.1	5.8
Tiny YOLOv3	4096 ∗ 4096	416 ∗ 416	41.1	23.2
The proposed improved YOLOv3	4096 ∗ 4096	416 ∗ 416	71.6	14.0

## Data Availability

All data can be obtained from the corresponding author upon request.
